# ESM1 Is a Promising Therapeutic Target and Prognostic Indicator for Esophageal Carcinogenesis/Esophageal Squamous Cell Carcinoma

**DOI:** 10.1155/2022/5328192

**Published:** 2022-07-27

**Authors:** Juan Li, Dong Yang, Cong Zhang, Sisi Wei, Ruinian Zhao, Suli Dai, Baoen Shan

**Affiliations:** ^1^Department of Intensive Care Unit, The Fourth Hospital of Hebei Medical University, Shijiazhuang, 050011 Hebei, China; ^2^Department of Emergency (Xiangjiang Hospital), The Third Hospital of Hebei Medical University, Shijiazhuang, 050051 Hebei, China; ^3^Research Center, The Fourth Hospital of Hebei Medical University, Shijiazhuang, 050011 Hebei, China

## Abstract

**Objective:**

Endothelial cell-specific molecule 1 (ESM1) has been implicated as an oncogene in several types of cancer. However, the potential role of ESM1 in esophageal carcinogenesis (ESCA)/esophageal squamous cell carcinoma (ESCC) is still unclear.

**Methods:**

The expression, function, and survival data of ESM1 were observed using a bioinformatics approach. Subsequently, the expression level of ESM1 in surgical esophageal tumors and adjacent normal tissues was detected by qRT–PCR and immunofluorescence. We further revealed protein expression by immunohistochemistry (IHC), which is related to the prognosis of patients with ESCC using survival analysis. In vitro, knockdown of ESM1 in KYSE150 and KYSE510 cell lines, colony formation assays, wound healing assays, and Transwell assays were performed.

**Results:**

ESM1 is significantly elevated in 12 of 20 types of human cancer. ESM1 is highly expressed in tumor tissue compared with adjacent normal tissue and was identified as a hub gene in ESCA. Clinical outcome endpoints of overall survival (OS), progression-free interval (PFI), and disease-specific survival (DSS) curves showed that patients whose ESM1 expression was high had a lower clinical survival rate. The ESM1 high-expression group has a certain correlation with clinical stage and grade. The IHC of ESM1 further demonstrated that the higher the expression was, the worse the N classification and pTNM stage in patients with ESCC, which had a distinctly poorer overall 5-year survival rate. Univariate analysis showed that age, N classification, pTNM stage, and ESM1 expression were all prognostic factors, although multivariate Cox regression analysis showed that only pTNM stage was an independent prognostic factor. In vitro, silencing ESM1 suppressed the proliferation, migration, and invasion of KYSE150 and KYSE510 cells.

**Conclusions:**

ESM1 is a hub gene in the initiation and progression of ESCA/ESCC that promotes the proliferation, migration, and invasion of esophageal cancer cells and may be a promising therapeutic target and prognostic indicator.

## 1. Introduction

Globally, for 204 countries and territories, the cancer burden was estimated to cause 23.6 million incident cancer cases and 10.0 million deaths, which has been provided by The Global Burden of Disease 2019 Cancer Collaboration (GBD2019) [1]. The International Agency for Research on Cancer (IARC) [2] reported updated data about the global cancer burden, indicating that it has risen to 28.4 million cases in 2040. Esophageal cancer ranks 7th in the incidence rate among malignancies globally and is 6th in overall mortality [2]. The pathological classification of esophageal carcinogenesis (ESCA) includes esophageal squamous cell carcinoma (ESCC) and adenocarcinoma, and 90% cases of esophageal cancer cases are ESCC [3]. Although surgery, chemotherapy, and targeted therapy have improved the prognosis of ESCC, the 5-year survival rate remains less than 20% [4, 5]. Therefore, the identification of new molecular biomarkers might provide further insights into the underlying molecular mechanisms affecting the occurrence and development of esophageal cancer and may have translational implications for biomarker identification and improving advanced therapies [3].

Human gene endothelial cell-specific molecule 1 (ESM1) cDNA was first cloned from a human umbilical vein endothelial cell cDNA library in the laboratory by Lassalle et al. in 1996 [6]. ESM1 is located on chromosome 5 at position q11.2. ESM1, a gene that encodes a soluble secretory proteoglycan, was also called endocan in 2001 [6, 7]. ESM1 is expressed in human vascular endothelial cells, hepatocytes, and renal tubular epithelial cells, and the function of ESM1 is mainly related to the inflammatory response, angiogenesis, and tumor cell growth [8–11]. Recently, ESM1 has been implicated in the tumorigenesis and development of multiple cancers, including colorectal cancer, epithelial ovarian cancer, head and neck cancer, and prostate cancer [12–15]. Although the role of ESM1 has been established in a previous study [16], little is known regarding the clinical and biological significance of ESM1 in ESCC.

Herein, this study intends to combine a bioinformatics approach and molecular biological experiments to verify ESM1 as the hub gene in esophageal cancer and thereby further identify the clinical and biological function as well as survival prognosis of ESM1 in ESCC.

## 2. Materials and Methods

### 2.1. Data Source and Differential Expression Analysis (DEGs)

The Cancer Genome Atlas (TCGA) (https://portal.gdc.cancer.gov/) online database [17] provides pancancer gene expression analysis of multiple cancer types. We searched for ESCC datasets from the Gene Expression Omnibus (GEO) database and downloaded GSE161533 (https://www.ncbi.nlm.nih.gov/geo/query/acc.cgi?acc=gse161533) (28 normal tissues, 28 paratumor tissues, and 28 tumor tissues). The R language limma software package was used to perform quantile standardization of RNA-seq data and identify differentially expressed genes (DEGs) (|logFC| > 1, *p* value < 0.05). The ggplot2 software package was used to construct a visual DEG volcano map and cluster analysis heatmap. Another ESCA dataset was derived from TCGA (162 tumor samples and 11 normal samples). DEGs were obtained by the R language edgeR package. Then, a visual DEG volcano map and cluster analysis heatmap were constructed.

### 2.2. Protein–Protein Interaction (PPI) Network Construction and Hub Gene Identification

A PPI network of hub genes was constructed using the online database search tool STRING (https://www.string-db.org/) [18], and a confidence score of ≥0.7 was set as the threshold. Protein nodes that did not interact with other proteins were removed. Furthermore, the PPI network was analysed to screen the significant modules and hub genes using Cytoscape (version: 3.8.0) [19]. The CytoHubba (version: 0.1) plug-in molecular complex detection (MCODE) [20] was used to screen the PPI network, and genes with degree > 10 were identified as hub genes.

### 2.3. Functional Enrichment Analysis and Construction of the Hub Gene-Pathway Network

The DEGs were subjected to Gene Ontology (GO) [21] and Kyoto Encyclopedia of Genes and Genomes (KEGG) enrichment analyses [22]. The DEGs in the biological process, cellular component, and molecular function categories were analysed using the online database tool DAVID (https://david.ncifcrf.gov) [23] to integrate the GO terms. The GO and KEGG pathway enrichment analysis diagrams of DEGs were plotted using the clusterProfler package of the R software. A hub gene-pathway network was constructed for DEGs using the web-based tool GeneCodis4 [24].

### 2.4. Clinical Survival and Prognosis Analysis

To explore survival analysis related to common clinical outcome endpoints and different clinical stages of ESCC according to gene expression level, TCGA database was used.

### 2.5. The Specimen Source

Tumor tissue specimens (confirmed by pathological diagnosis) and matched adjacent normal tissue specimens (at least 5 cm away from the tumor margin) were collected from 49 patients with ESCC who underwent surgical resection from December 2019 to December 2020 in the Department of Thoracic Surgery, The Fourth Hospital of Hebei Medical University. Additional paraffin-embedded tumor samples were selected from 83 patients undergoing surgery in our hospital who were then diagnosed with ESCC by the pathology department from January 2013 to July 2016. This study was approved by the Ethics Committee of the Fourth Hospital of Hebei Medical University and accepted by the patient informed consent. Patients whose age was less than 18 years and who underwent preoperative radiotherapy, chemotherapy, or biological therapy were excluded. The 83 cases of postoperative TNM staging were performed according to the standard of international TNM staging (8th edition) formulated by the International Union Against Cancer and the United States Joint Commission on Cancer (UICC/AJCC) [25]. The overall survival of 83 patients was defined as the endpoint from the date of surgery to death. Follow-up assessments were performed for the first overall 5-year survival rate after surgery.

### 2.6. Immunofluorescence (IF) and Immunohistochemistry (IHC)

The expression of ESM1 was detected by immunofluorescence staining of 26 cases of esophageal carcinoma and matched adjacent normal tissue. Tissue sections were incubated with anti-ESM1 rabbit polyclonal antibody (Abcam, No.: ab103590) at 37°C for 60 min or at 4°C overnight and then with tritC-conjugated anti-rabbit immunoglobulin (Abcam, No.: ab150081) at room temperature for 60 min. Finally, the sections were photographed under a fluorescence microscope, and the mean fluorescence intensity was calculated. Another a group of sections were derived from 83 corresponding paraffin-embedded tumor samples, in which haematoxylin-eosin (HE) staining was performed for tumor diagnosis and the ESM1 was further detected by IHC (streptavidin-peroxidase method). All sections were assessed by two experienced pathologists independently. The immunoreactivity was defined as brown in the cytoplasm of tumor cells. The ESM1 expression level was evaluated by the immunoreactive score (IRS), which is equal to the percentage of positive cells (PPs) multiplied by the staining intensity (SI) [26]. PP was scored as follows: 0 (no positive tumor cell), 1 (<10%), 2 (10-50%), 3 (51-80%), and 4 (>80%). SI was scored as follows: 0 (negative), 1 (weak), 2 (moderate), and 3 (strong staining). Five random visual fields from different areas of each slide were viewed. Scores of at least 4 points were defined as high ESM1 expression.

### 2.7. Knockdown Expression of ESM1 in ESCC Cell Lines

Small interfering RNAs (siRNAs, si-NC, si-ESM1#1, si-ESM1#2, and si-ESM1#3) were purchased from Shanghai GenePharma Co., Ltd. KYSE150 and KYSE510 cells were obtained from the Shanghai Institute for Biological Sciences and cultured with RPMI-1640 medium (Gibco, No.: 11875093) containing 10% fetal bovine serum (FBS), 100 U/ml penicillin, and 100 *μ*g/ml streptomycin at 37°C and 5% CO_2_. When the cell density reached 80%, the cells were digested with trypsin and subcultured. Then, the cells in logarithmic growth phase were harvested, and according to the guidelines of the manufacturer, KYSE150 and KYSE510 cells were transiently transfected with 3 *μ*l si-ESM1 #1 (5′-3′: justice chain: GGU GAA GAG UUU GGU AUC UTT and antisense chain: AGA UAC CAA ACU CUU CAC CTT), si-ESM1#2 (5′-3′: justice chain: GGA GAU GGC AAU AUU GUG ATT and antisense chain: UCA CAA UAU UGC CAU CUC CTT), and si-ESM1 #3 (5′-3′: justice chain: CCC GUA AUG AGG AAA UGG UTT and antisense chain: ACC AUU UCC UCA UUA CGG GTT). These two cell lines were divided into the interference groups (si-ESM1#1 group, si-ESM1#2 group, and si-ESM1#3 group) and the negative control group (si-NC group).

### 2.8. RNA Extraction and qRT–PCR

RNA was extracted from the transfected KYSE150 and KYSE510 cells and tissue specimens according to routine laboratory procedures, and the RNA concentration was detected. Reverse transcription was performed according to the instructions of the purchased reverse transcription kit (Invitrogen, No. 4368814) (reaction conditions: 37°C for 15 min, 85°C for 5 sec, and 4°C + ∞). Then, the program was set up on the machine to conduct PCR, and finally, the reaction results were derived, and the data were analysed using the 2-△△Ct statistical method. Primer sequences were purchased from Shanghai Generay Biotech Co., Ltd, as shown in Table 1 below.

### 2.9. Monoclonal Proliferation Assay

At 48 hr after transfection, the cells were collected, digested with trypsin, and counted. They were cultured in a 37°C incubator for approximately 2 weeks until there were visible clonal clusters. After the medium was discarded, the cells were washed with PBS 3 times, fixed with methanol for 15 min, air dried, and stained with crystal violet for 30 min. After drying, the cells were scanned and photographed, and the visible clonal clusters were counted.

### 2.10. Wound Healing Assay and Detection of Migration and Invasion in ESCC Cells by Transwell Assay

The cells (1 × 10^5^) were seeded into 6-well plates. When the cell density reached 100%, the well was scratched vertically along the central axis using a 1 ml pipette tip, and the shedding cells were washed away. At 0 hr, 24 hr, and 48 hr, the wound healing status was photographed under a light microscope, and then, the percentage of the wound area was calculated.

Migration assay: after transfection into KYSE150 and KYSE510 cells (2 × 10^5^ cells/ml), 200 *μ*l of cell suspension without serum and 600 *μ*l of media with 10% FBS were added into the upper and lower Transwell chambers, respectively, cultured for 24 hr, fixed with methanol, and stained with crystal violet. Then, the number of migrating cells was observed. Invasion assay: a protocol similar to the migration assay was used except that the Transwell units were precoated with 200 *μ*g/ml Matrigel and incubated overnight.

### 2.11. Statistical Analysis

The SPSS 21.0 software was used to analyse the experimental data. Continuous variables with a normal distribution are presented as the mean ± standard deviation (*x̅*±*s*), and nonnormal variables are reported as the median (interquartile range (IQR)). Data were compared by *T* test, one-way ANOVA, Mann-Whitney *U* test, and Wilcoxon rank sum test. A chi-square test or Fisher's exact test was used for categorical variables. Survival analysis was performed using the Kaplan-Meier method with the log-rank test. Univariate and multivariate Cox regression analyses were conducted to analyse prognostic factors. *p* < 0.05 was considered statistically significant.

## 3. Results

### 3.1. General Overexpression of ESM1 in Multiple Types of Human Cancer

TCGA pancancer gene expression analysis indicated that the expression of ESM1 is significantly elevated in 12 of 20 types of human cancer (see Figure 1(a)). In TCGA database of ESCA, compared with 11 normal tissues, ESM1 was highly expressed in 162 tumor tissues (*p* < 0.001, see Figure 1(b)), and ESM1 expression in 11 of 162 tumor tissues was also higher than that in 11 paired adjacent tissues (*p* < 0.001, see Figure 1(c)). Similarly, we observed data from GEO-GSE161533 in which the expression level of ESM1 was remarkably higher in tumors than in normal and paratumor tissues (28 tumor, 28 normal, and 28 paired paratumor samples, *p* < 0.001) (see Figures 1(d)–1(f)).

### 3.2. Identification of DEGs

The data were screened in GEO-GSE161533 (*p* < 0.05 and |logFC| > 1). There were 1219 DEGs between ESCA and normal tissue, comprising 559 upregulated DEGs and 660 downregulated DEGs. ESM1 is in the upregulation zone (see Figure 2(a)). The heatmap showed that ESM1 is an upregulated DEG in tumor tissue (see Figure 2(c)). Derived from another TCGA dataset, there were 482 DEGs between ESCA and normal tissue, including 354 upregulated DEGs and 128 downregulated DEGs. ESM1 is also in the upregulation zone (see Figure 2(b)). Their corresponding heatmap showed that ESM1 is an upregulated DEG in tumor tissue (see Figure 2(d)).

### 3.3. Construction of the PPI Network, Hub Gene Screening, Functional Enrichment Analysis, and Hub Gene-Pathway Network

The intersection of 144 DEGs from the GSE161533 and TCGA datasets is shown by a Venn diagram (see Figure 3(a)). Then, a PPI network of 144 DEGs was obtained using the Cytoscape software. Red and green represent upregulated and downregulated genes, respectively, in which ESM1 is significantly upregulated (see Figure 3(b)). The PPI network was screened by the CytoHubba software, and genes with a degree > 10 were identified as hub genes (see Figure 3(d)). As Table 2 shows, the score of ESM1 is higher than that of the other genes. These ten hub genes may be involved in the interaction that contributes to the carcinogenic process of ESCA. GO functional enrichment analysis of 144 DEGs suggested their potential biological processes, which involve the cell cycle, cell division, inflammatory response, cell-cell signalling, chemotaxis, chromosome segregation, chemokine-mediated signalling pathway, etc. (see Figure 3(e)). KEGG and the hub gene-pathway network indicated a few signalling pathways, such as cytokine-cytokine receptor interaction, the IL-17 signalling pathway, TNF signalling pathway, transcriptional misregulation in cancer, and chemokine signalling pathway (see Figures 3(c) and 3(f)). ESM1 may be involved in the initiation and progression of ESCA by the above potential signalling pathways.

### 3.4. Clinical Outcome Endpoints of Overall Survival (OS), Progression-Free Interval (PFI), Disease-Specific Survival (DSS), and Disease-Free Interval (DFI)

TCGA-related survival data were downloaded for Kaplan-Meier survival analysis, and the OS, PFI, DSS, and DFI curves were plotted. They are four common clinical outcomes used in cancer research. As Figure 4 (see Figures 4(a)–4(c)) shows, compared with the ESM1 low-expression group, the OS, PFI, and DSS were shorter in the ESM1 high-expression group (*p* < 0.05). All hazard ratios greater than 1 indicate that ESM1 might predict clinical prognosis in ESCA. However, in DFI, the outcome is the opposite, which might be due to a small sample size (see Figure 4(d)).

### 3.5. Clinical Stage and Survival Probability of High ESM1 Expression

Clinical data regarding ESCA were derived from TCGA dataset. Compared with the normal healthy control, the ESM1 expression level in patients with clinical stage I, stage II, and stage III disease increased (*p* < 0.01). There was no difference in overall survival probability between patients with different stages because of the small sample size (see Figure 5(a)). Regarding T stage, the ESM1 expression level in patients with T1-T4 disease was higher than that in normal healthy controls (*p* < 0.05). Furthermore, patients with T4 stage had the lowest survival rate (*p* = 0.012) (see Figure 5(b)). Compared with normal healthy controls, the more lymph node metastases there were, the higher the ESM1 expression, except at the N2 stage, which might be due to only 4 patients (*p* < 0.01). As lymph node metastasis increased, the prognosis gradually worsened (*p* = 0.0039) (see Figure 5(c)). ESM1 expression was higher in patients with involvement of peripheral organs than in normal healthy controls, which have poorer outcomes (*p* = 0.018) (see Figure 5(d)). Thus, ESM1 may be a promising clinical prognostic indicator.

### 3.6. The Expression of ESM1 Was Detected by qRT–PCR, IF, and IHC

Compared with matched adjacent normal tissue, the mRNA expression level of ESM1 in esophageal carcinoma was significantly elevated. The results showed that the median expression level of ESM1 in cancer tissues was 1.37 (0.40-6.44), and in adjacent normal tissue, it was 0.34 (0.12-1.56) (*p* = 0.01) (see Figure 6(a)). The protein expression level, namely, endocan, was remarkably expressed in esophageal cancer tissues and weakly expressed in adjacent normal tissue by IF, and the mean fluorescent intensity of ESM1 in esophageal carcinoma was also elevated compared with matched adjacent normal tissue (*p* < 0.01) (see Figure 6(b)). HE staining was performed for tumor diagnosis (see Figures 6(c) and 6(d)). IHC staining showed that the immunoreactivity of ESM1 was primarily expressed in the cytoplasm of tumor cells and not in normal esophageal squamous epithelial cells (see Figure 6(e)). Regarding immunoreactive scores, at least 4 points were defined as high ESM1 expression. Low: −~+; high: ++~+++ (see Figures 6(f)–6(i)).

### 3.7. Higher ESM1 Expression Was Associated with Clinicopathological Features and Poor Prognosis in 83 Patients with ESCC

ESM1 expression is closely related to the N classification and pTNM stage (see Table 3). Linear association showed that the higher the ESM1 expression was, the poorer the N classification (*χ*^2^ = 7.775, *p* = 0.005). The ESM1 expression level was significantly higher in pathological TNM stage III+IV than in stage I+II (*χ*^2^ = 4.219, *p* = 0.04). Furthermore, Kaplan-Meier survival analysis demonstrated that patients with higher ESM1 expression had a distinctly poorer overall 5-year survival rate (*p* = 0.036) (see Figure 6(j)). Univariate analysis showed that age (HR = 4.287, 95% CI 1.262-14.564, and *p* = 0.02), N classification (HR = 2.055, 95% CI 1.321-3.197, and *p* = 0.001), pTNM stage (HR = 2.663, 95% CI 1.543-4.594, and *p* ≤ 0.001), and ESM1 expression (HR = 2.425, 95% CI 1.027-5.726, and *p* = 0.043) were prognostic factors, while multivariate Cox regression analysis showed that only pTNM stage (HR = 2.031, 95% CI 1.039-3.972, and *p* = 0.038) is an independent prognostic factor (see Table 4).

### 3.8. Effect of Silencing the ESM1 Gene on the Proliferation, Migration, and Invasion of ESCC Cells

Given ESM1 overexpression in ESCA, small interfering RNA (siRNA) was used to knockdown the gene by transient transfection, and then, the biological function of ESM1 was observed. qRT–PCR results showed that compared with the si-NC group, the mRNA relative expression levels of ESM1 in the interference group were distinctly downregulated. The knockdown efficiency of the ESM1 gene was more significant in si-ESM1#2 and si-ESM1#3 (*p* < 0.05; *p* < 0.01) (see Figure 7(a)). The effect of silencing the ESM1 gene on the proliferation ability of esophageal cancer cells was assessed through a monoclonal proliferation assay. The number of colonies formed in KYSE150 and KYSE510 cells was distinctly smaller in the si-ESM1#3 group than that in the si-NC group (*p* < 0.01; *p* < 0.05) (see Figure 7(b)). The results of the wound healing assay revealed that at 24 hr and 48 hr after scratching, the percentage of the wound area of KYSE150 and KYSE510 cells was significantly increased in the si-ESM1#2 group and si-ESM1#3 group compared with the si-NC group, suggesting that the migratory rate of cells was obviously reduced (see Figure 7(c)). Similarly, the results of migration and invasion assays showed that the numbers of migrating cells and those passing through the basement membrane were apparently smaller in the si-ESM1#2 group and in the si-ESM1#3 group than in the si-NC group (*p* < 0.05; *p* < 0.01) (see Figure 7(d)). ESM1 silencing inhibited the migration and invasion of esophageal cancer cells.

## 4. Discussion

Due to the lack of specific early symptoms, obvious signs, and early diagnostic markers, patients with esophageal cancer are usually in later stages at the time of treatment, and their prognosis is unsatisfactory [27]. Therefore, identifying more molecular markers for prognostic estimation is important for prolonging the survival time of patients with esophageal cancer. Recently, ESM1 has been shown to have a high expression level in numerous types of cancer [12–15], suggesting that it may be a potential biomarker for the diagnosis and treatment of different cancers.

As seen from analysis of the GSE161533 and TCGA database, ESM1 is notably elevated in 12 of 20 types of human cancer, including ESCA. Our qPCR and IF results also demonstrate that the gene and protein expression of ESM1 are higher in ESCC than adjacent normal tissues. We subsequently explored the biological function of ESM1 in esophageal cancer cells. Malignancies have important biological characteristics, such as malignant proliferation, invasion, and metastasis [28, 29]. In this study, the effects of silencing ESM1 on the proliferation, migration, and invasion of esophageal cancer cells were observed by a monoclonal proliferation assay, wound healing assay, and Transwell assay, respectively. The number of colonies formed in KYSE150 and KYSE510 cells was distinctly smaller in the si-ESM1#2 group and si-ESM1#3 group than that in the si-NC group. At 48 hr after scratching, the scratch area of KYSE150 and KYSE510 cells was significantly larger in the si-ESM1#2 group and si-ESM1#3 group than that in the si-NC group, suggesting that the migration distance of tumor cells towards the center of the scratch was reduced. Similarly, the Transwell assay showed that the migration and invasion were remarkably lower in the si-ESM1#2 group and si-ESM1#3 group than in the si-NC group. The above findings demonstrate that silencing ESM1 suppresses the proliferation, migration, and invasion of esophageal cancer cells. Cui et al. [16] have also confirmed that knockdown of ESM1 inhibited proliferation and migration, while overexpression promoted them in KYSE70 cells. The above results show that ESM1 may perform a carcinogenic action in ESCC.

The name of the ESM1 gene product is called endocan, which is composed of a 165 amino acid core polypeptide chain and a DS chain covalently bound to the serine residue at position 137 of the core polypeptide chain. Endocan is secreted by endothelial cells into the blood and is highly expressed in some tumor cells. There are two major sites associated with tumors, termed DS chains and phenylalanine-rich regions, which are located at positions 113-118 of the core polypeptide chain [6, 7, 30]. Endocan is regulated by proinflammatory molecules and proangiogenic growth factors. TNF-*α* and IL-1 can lead to the upregulation of endocan, while it can be downregulated by IFN-*γ* [31, 32]. Data derived from the hub gene-pathway network indicated that the IL-17 signalling pathway, TNF signalling pathway, NF-*κ*B, JAK-STAT signalling pathway [16], and cytokine-cytokine receptor interaction may be involved in the progression of ESCA.

The GSE161533 and TCGA database analyses showed that ESM1 was not only a hub gene and played a crucial role in the initiation and development of ESCA but also correlated with a low survival rate, including OS, PFI, and DSS, as well as clinical stage and grade. To date, ESM1 expression in IHC of ESCC has never been reported. In this study, we found that ESM1 was predominantly highly expressed in the cytoplasm of tumor cells and further demonstrated that the higher the ESM1 expression level was, the worse the N classification and pTNM stage in 83 patients with ESCC, which had a distinctly poorer overall 5-year survival rate. Subsequently, univariate analysis showed that age, N classification, pTNM stage, and ESM1 expression (HR = 2.425, 95% CI 1.027-5.726, and *p* = 0.043) were all prognostic factors, although multivariate Cox regression analysis showed that only pTNM stage was an independent prognostic factor. Perhaps the number of enrolled patients was relatively small. Thus, it is necessary to further expand the sample quantity to better explore the role of ESM1 in ESCC.

In addition, several studies have shown high ESM1 expression not only in cancer tissues [33] but also in serum [34, 35] and pleural effusion [36]. ESM1 is a potential prognostic biomarker in corresponding cancer. In future studies, combining gene expression and serum levels of ESM1 together to predict cancer prognosis could be a potential research direction.

## 5. Conclusions

In conclusion, the expression and prognostic significance of ESM1 in esophageal cancer were comprehensively analysed using online databases in this study, and its high expression and potential clinical value in esophageal cancer were revealed, providing a theoretical basis for understanding the role of ESM1 in ESCA. Bioinformatics analysis and experimental results proved that ESM1 is a hub gene and that silencing ESM1 can significantly inhibit the proliferation, migration, and invasion of esophageal cancer cells, providing a preliminary scientific basis for future research on clinical prognostic biomarkers and/or targeted therapy. However, the sophisticated and precise regulatory mechanism of ESM1 in esophageal cancer needs further study.

## Figures and Tables

**Figure 1:** The expression of ESM1 in TCGA pancancer gene expression analysis and GSE161533 GEO database. (a) ESM1 is significantly highly expressed in 12 of 20 types of human cancer, including ESCA. Red and blue represent tumor (*T*) and normal (*N*) tissues, respectively. (b) ESM1 is distinctly highly expressed in ESCA (*T* = 162, *N* = 11). (c) ESM1 is highly expressed in tumors compared with the paired normal tissue (*T* = 11, *N* = 11). (d–f) ESM1 was remarkably highly expressed in ESCA tumors compared with normal and/or the paired tissues (*T* = 28, *N* = 28, and para-*T* = 28). ^∗^*p* < 0.05, ^∗∗^*p* < 0.01, and ^∗∗∗^*p* < 0.001.

**Figure 2:** Volcano plot and heatmap of DEGs between ESCA and normal or paratumor tissue samples from the GSE161533 and TCGA datasets. (a, b) Orange represents the upregulated DEGs. ESM1 is an upregulated DEG. (c, d) Blue and red represent upregulated and downregulated DEG, respectively. ESM1 is an upregulated DEG in tumor tissue.

**Figure 3:** PPI network, hub genes, functional enrichment analysis, and hub gene-pathway network. (a) The Venn diagram shows 144 DEGs that were commonly upregulated and downregulated between the two datasets. (b) Red and green represent upregulation and downregulation of the PPI network of the 144 DEGs, respectively. (c) Hub gene and related pathway network. Red, green, and pink represent upregulated, downregulated genes, and pathways, respectively. (d) ESM1 is a hub gene located in the top among the top 10 DEGs. (e, f) GO and KEGG presentation of 144 DEGs. The abscissa represents the larger enrichment ratio and the higher enrichment degree. Likewise, red represents a higher enrichment degree, and black represents a larger circle indicating a more enriched gene.

**Figure 4:** Survival analysis curve of the ESM1 high-expression and low-expression groups. Red and blue represent the ESM1 high- and low-expression groups, respectively. (a) The higher expression of ESM1, the worse prognosis of OS (HR = 1.19, 95% CI 1.01-1.42, and *p* < 0.0001), (b) PFI (HR = 1.13, 95% CI 0.96-1.33, and *p* = 0.033), and (c) DSS (HR = 1.34, 95% CI 1.11-1.62, and *p* < 0.0001). (d) DFI was longer in the ESM1 high-expression group.

**Figure 5:** Correlation between ESM1 expression and clinical stage/grade as well as overall survival probability of ESCC patients. Data derived from TCGA dataset. (a) ESM1 expression levels in patients with clinical stage I, stage II, and stage III disease were significantly higher than those in healthy controls. The prognosis of the three groups was not significantly different. (b) Regarding T stage, the ESM1 expression level in patients with T1-T4 stage disease was higher than that in normal healthy controls. T4 patients had the lowest survival rate. (c) Compared with normal healthy controls, the more lymph node metastases there were, the higher the ESM1 expression, except at the N2 stage. The number of metastatic lymph nodes correlates inversely with OS. (d) ESM1 expression was higher in patients with involvement of peripheral organs. The prognosis of patients with distant organ metastasis is poor. ^∗^*p* < 0.05, ^∗∗^*p* < 0.01, and ^∗∗∗^*p* < 0.001.

**Figure 6:** ESM1 was highly expressed in esophageal carcinoma and the corresponding survival rate. (a) The mRNA expression of ESM1 was detected by qRT–PCR in adjacent normal tissue and esophageal cancer. (b) ESM1 protein expression was detected by IF of adjacent normal tissue and esophageal cancer tissue. Scale bar equals 50 *μ*m. Blue indicates cell nuclei, and green indicates ESM1. The mean fluorescence intensity in adjacent normal tissue and esophageal cancer was 1.00 ± 1.07 and 3.29 ± 0.17, respectively. (c) Normal squamous epithelium adjacent to carcinoma (HE×100). (d) Esophageal squamous cell carcinoma (HE×200). (e) Negative expression of ESM1 in squamous epithelium adjacent to carcinoma (IHC SP×100). (f–i) ESM1 is (-)(+)(++)(+++) in ESCC (IHC SP×200). (j) Patients whose ESM1 IHC high-expression had a lower 5-year overall survival rate (*p* = 0.036). ^∗^*p* < 0.05 and ^∗∗^*p* < 0.01.

**Figure 7:** ESM1 promoted the proliferation, migration, and invasion of esophageal cancer cells. (a) KYSE150 and KYSE150 cells were transfected with siRNA, and the expression of ESM1 was detected by qRT–PCR. The knockdown efficiency of the ESM1 gene was more significant in si-2 and si-3. (b) Knockdown of ESM1 inhibited the colony formation ability of KYSE150 and KYSE510 cells. (c) Wound healing assay showed the effect of silencing ESM1 on cell mobility. (d) Transwell assays were used to detect the effect of silencing ESM1 on migration and invasion. ^∗^*p* < 0.05 and ^∗∗^*p* < 0.01.

**Table 1:** Primer sequences.

Gene	Primer sequences
ESM1	F: GCCTGAGACTGTGCGGTAG
	R: CTGGGAAACATGAAGAGCG
GAPDH	F: GGACCTGACCTGCCGTCTAG
	R: GTAGCCCAGGATGCCCTTGA

**Table 2:** Top 10 genes in the PPI network ranked by degree method.

Rank	Gene name	Score
1	ESM1	32
2	MMP9	18
2	CXCL1	18
4	CXCL10	15
4	CCL20	15
6	CXCL5	14
7	SPP1	10
7	IL11	10
9	MMP3	9
9	IL36G	9

**Table 3:** The associations between ESM1 expression and clinicopathological characteristics in 83 ESCC patients. ^∗^*p* < 0.05 and ^∗∗^*p* < 0.01.

Characteristics	*n*	ESM1 expression		*χ* ^2^	*p*
		Low (*n*(%))	High (*n*(%))		
All	83	54 (65.1)	29 (34.9)		
Age (year)				2.263	0.132
<60	32	24 (44.4)	8 (27.6)		
≥60	51	30 (55.6)	21 (72.4)		
Gender				0.813	0.367
Male	54	37 (68.5)	17 (58.6)		
Female	29	17 (31.5)	12 (41.4)		
Tumor size (cm^3^)				1.116	0.291
<5	10	8 (14.8)	2 (6.9)		
≥5	73	46 (85.2)	27 (93.1)		
T classification				3.009	0.390
Tis	1	1 (1.9)	0 (0)		
T1	3	2 (3.7)	1 (3.4)		
T2	16	13 (24.1)	3 (10.3)		
T3	63	38 (70.4)	25 (86.2)		
N classification				7.775	0.005^∗∗^
N0	44	35 (64.8)	9 (31.0)		
N1	31	15 (27.8)	16 (55.2)		
N2	6	4 (7.4)	2 (6.9)		
N3	2	0 (0)	2 (6.9)		
M classification				—	—
M0	83	54	29		
M1	0	0	0		
pTNM stage				4.219	0.04^∗^
I+II	47	35 (64.8)	12 (41.4)		
III+IV	36	19 (35.2)	17 (58.6)		
Pathological differentiation				5.608	0.132
High differentiation	8	8 (14.8)	0 (0)		
Middle differentiation	58	36 (66.7)	22 (75.9)		
Low differentiation	16	9 (16.7)	7 (24.1)		
Undifferentiated	1	1 (1.9)	0 (0)		
Tumor embolus				0.522	0.47
Negative	78	50 (92.6)	28 (96.6)		
Positive	5	4 (7.4)	1 (3.4)		

**Table 4:** Univariate and multivariate Cox regression analyses of overall survival in 83 patients with ESCC. ^∗^*p* < 0.05 and ^∗∗^*p* < 0.01.

Parameter	Overall survival			
	Univariate analysis		Multivariate analysis	
	HR (95% CI)	*p*	HR (95% CI)	*p*
Age	4.287 (1.262-14.564)	0.02^∗^	3.225 (0.937-11.095)	0.063
Gender	0.738 (0.311-1.751)	0.49	--	--
Tumor size	1.526 (0.355-6.556)	0.57		
T classification	3.155 (0.817-12.181)	0.095		
N classification	2.055 (1.321-3.197)	0.001^∗∗^	1.38 (0.616-3.094)	0.434
pTNM stage	2.663 (1.543-4.594)	≤0.001^∗∗^	2.031 (1.039-3.972)	0.038^∗^
Pathological differentiation	1.468 (0.697-3.094)	0.312	--	--
Tumor embolus	2.223 (0.517-9.555)	0.283		
IHC score-ESM1	2.425 (1.027-5.726)	0.043^∗^	1.506 (0.634-3.578)	0.353

## Data Availability

The data and materials in the current study are available from the corresponding author on reasonable request.
